# Curcumin Elevates microRNA-183-5p via Cathepsin B-Mediated Phosphatidylinositol 3-Kinase/AKT Pathway to Strengthen Lipopolysaccharide-Stimulated Immune Function of Sepsis Mice

**DOI:** 10.1155/2022/6217234

**Published:** 2022-07-30

**Authors:** Yanan Liu, LiZhi Feng, Guo Hou, Lan Yao

**Affiliations:** Department of Critical Care Medicine, Renmin Hospital of Wuhan University, Wuhan, Hubei Province 430030, China

## Abstract

Curcumin (Cur), a natural polyphenol compound, has been testified to modulate innate immune responses and also showed *anti*-inflammatory properties. Nevertheless, the mechanism was still poorly unknown, especially regarding Cur-modulated microRNAs (miRNAs) under the inflammatory response. CD39^+^ regulatory T cells (Tregs) were provided with distinct immunosuppressive action and exerted a critical role in the modulation of immune balance in sepsis. Nevertheless, the impact of Cur on the immune function of sepsis mice has not been reported. In this study, the influence of Cur on the inflammatory response and immune function of sepsis mice via augment of miR-183-5p and Cathepsin B (CTSB)-mediated phosphatidylinositol 3-kinase (PI3K)/AKT pathway was explored. Adoption of 20 mg/kg Cur was for gavage. In the meantime, injection of plasmid vectors of interference with miR-183-5p or CTSB was into the tail vein. Intraperitoneal injection of lipopolysaccharide (10 mg/kg) was to stimulate model of sepsis mice. Histopathological changes of sepsis mice were observed. The contents of tumor necrosis factor-*α* and Interleukin (IL)-1*β* and IL-6 in serum of mice were examined. Detection of alanine aminotransferase, aspartate aminotransferase (AST), urea nitrogen (BUN), and creatinine in serum of mice was performed. Test of the percentage of CD39^+^ Tregs in tail venous blood of mice was implemented. Examination of miR-183-5p, CTSB, and PI3K/AKT was performed. The targeting of miR-183-5p and CTSB was detected. Cur was available to ameliorate the histological damage, to reduce the content of inflammatory factors, AST, and BUN, and to decline the percentage of CD39^+^ Tregs in tail venous blood of sepsis mice. Elevated miR-183-5p or silenced CTSB was available to further enhance the protection of Cur. Cur was available to accelerate miR-183-5p, which negatively modulated CTSB and Cur-mediated PI3K/AKT pathway via the miR-183-5p/CTSB axis to restrain inflammation of sepsis mice and enhance its immune function.

## 1. Introduction

Sepsis, a systemic inflammatory response syndrome caused via infection, influences millions of people worldwide every year with its growing incidence [1]. It is characterized via the massive release of cytokines and other mediators, thereby leading to the maladjustment of immune response and is supposed to result in organ injury and death [2]. Presently, it is broadly recognized that the occurrence of sepsis covers the initial immune activation phase and the subsequent chronic immunosuppression stage, and these two stages occur simultaneously, resulting in immune cell death [3]. Nevertheless, there is no explicit treatment for sepsis, while survivors also suffer from long-term immunosuppression and infection with an elevated recurrence rate [4]. Consequently, it is urgent to develop brand-new immunotherapy drugs for the therapy of sepsis.

Curcumin (Cur), the critical active component of turmeric, has been broadly explored for its multiple pharmacological activities, covering *anti*-tumor, *anti*-inflammatory and antioxidant properties [5]. Cur has been testified to be conducive to diversified diseases, for instance, Cur exerts an *anti*-inflammatory and antioxidant role in arsenic-stimulated liver and kidney injury via repressing mitogen-activated protein kinases/NF-*κ*B and activating Nrf2 pathways [6]. Cur constrains the malignant progression of nonsmall cell lung cancer via modulating the circ-PRKCA/miR-384/ITGB1 pathway [7]. Presently, numerous studies have testified that Cur is provided with a latent therapeutic action in sepsis. For instance, Cur ameliorates metabolic parameters during experimental sepsis via constraining the release of inflammatory cytokines and heat shock protein 70 [8]. Cur suppresses oxidative stress-associated inflammation via phosphatidylinositol 3-kinase (PI3K)/AKT and NF-*κ*B related signaling, thereby alleviating lipopolysaccharide (LPS)-stimulated sepsis and liver failure [9]. Cur with the ability of modulating the immune response of sepsis has been broadly testified, while its specific action mechanism has not been completely illuminated, particularly regarding Cur-modulated miRNA in the inflammatory response [10].

MicroRNA (miRNA) is a group of short single-stranded noncoding RNAs with about 18–22 nucleotides in length, lacking potential of protein coding, but it is available to modulate gene via repressing the translation or transcription of its target mRNA [11]. They implicate in almost all cell activities, covering cell growth, differentiation, development, and apoptosis [12]. Additionally, they are also associated with multiple diseases, covering cancer [13], immune-related diseases [14], neurological diseases [15], and cardiovascular diseases [16]. Numerous researches have clarified that miRNA exerts a crucial action in the occurrence and progression of sepsis. For instance, miRNA-133a aggravates the inflammatory response of sepsis via targeting sirtuin-1 [17]. Elevated miR-223 stimulates M2 macrophages and attenuates LPS-induced sepsis via changes of glycolysis [18]. Nevertheless, the role of numerous miRNAs in sepsis has not been completely explicit and further exploration should be performed. The study was to explore the influence of Cur on the immune function of sepsis mice and its latent mechanism and further analyze the interaction of Cur with miR-183-5p.

## 2. Materials and Methods

### 2.1. Model of Sepsis Mouse

This study was conducted in line with the institutional guidelines for animal care and use formulated via the Animal Care Committee of Renmin Hospital of Wuhan University. A batch of 8-week-old male C57BL/6 mice with weight of 21 ± 2 g was purchased (Shanghai Lab. Animal Research Center). All mice were kept free of specific pathogens and subjected to a 12-h light/dark cycle. In animal experiments, intraperitoneal injection of LPS (10 mg/kg) was to construct model of sepsis mice. Random division of C57BL/6 mice was into 7 groups with 6 animals in each group, as follows. The Sham: intraperitoneal injection with the same amount of normal saline; the LPS : intraperitoneal injection with LPS (10 mg/kg); the Cur : LPS + Cur (20 mg/kg); the Agomir negative control (NC) : LPS + Cur + agomir NC; the miR-183-5p agomir: LPS + Cur + miR-183-5p agomir; the si-NC : LPS + Cur + si-NC; the si-cathepsin B (CTSB) : LPS + Cur + si-CTSB. Mice were given 20 mg/kg Cur in gavage for 3 d; in the meantime, injection of plasmid vectors of interference with miR-183-5p or CTSB (10 nM per 20 g weight) (Ribo Biotechnology, Guangzhou, China) was into the tail vein. Then, intraperitoneal injection of LPS (10 mg/kg) was to stimulate the model of sepsis mice, and euthanasia was performed 16 h later.

### 2.2. Determination of Serum Biochemical Indexes

Determination of serum of alanine aminotransferase (ALT), aspartate aminotransferase (AST), urea nitrogen (BUN), and creatinine was via commercial kits (BioVision, Milpitas, California). Contents of tumor necrosis factor-*α* (TNF-*α*), interleukin (IL)-1*β*, and IL-6 in the serum was also determined via a commercial enzyme-linked immunosorbent assay kit (BioVision). In this paper, the effects of Cur on kidney and liver functions of septic mice were studied. The above serum indicators met the needs of this experiment.

### 2.3. Flow Cytometry

After taking tail vein blood samples, centrifugation at 800 rpm and removal of the supernatant were carried out. Then, addition of erythrocyte lysate was performed and the tube was kept for 5 min; centrifugation at 800 rpm was further again done. After discarding the supernatant, rinse of the cells was done twice with phosphate buffered saline (PBS) and suspension was performed again with a cell density adjusted to 1 × 10^6^/mL. Addition of antibodies *anti*-CD4-fluorescein isothiocyanate, *anti*-CD25-PE, *anti*-CD127-PerCP, and *anti*-CD39-APC (BD Pharmingen Corporation) was implemented and the test tube was incubated. A certain percentage of CD39^+^ regulatory T cells (Tregs) was analyzed adopting BD FACSCalibur system with FlowJo software. Definition of Tregs was as CD4^+^ CD25^+^ CD127^−^ lymphocytes. Percentage of CD39^+^ Tregs = (CD39^+^ Tregs count/total number of Tregs cells) × 100%.

### 2.4. Hematoxylin-Eosin (HE) Staining

Euthanasia of the mice was inhalation of CO_2_; kidneys and livers were taken out, and fixation was with 10% formalin for histological examination. Staining of paraffin-embedded tissue sections (7 *μ*m) was with HE. The sections were observed under a microscope (Olympus, Tokyo, Japan).

### 2.5. TdT-Mediated dUTP-Biotin Nick End-Labeling (TUNEL) Staining

The histopathological sections were dewaxed and incubated with protease K. Sections were stained adopting the terminal deoxynucleotidyl transferase dUTP nick end labeling (TUNEL) kit (Biovision, USA), and the cell nucleus was stained with 4′, 6-diamidino-2-phenylindole, and they were observed under the fluorescence microscope (ECLIPSE FNl, Nikon, Tokyo, Japan). Apoptotic cells were fluorescent green, while nuclei were blue.

### 2.6. Reverse Transcription Quantitative Polymerase Chain Reaction (RT-qPCR)

Extraction of total RNA was performed adopting TrizolReagent (Sigma–Aldrich). Synthesis of a complementary DNA (cDNA) which was implemented adopting the cDNA reverse transcription kit with high capacity (ThermoFisher Scientific). The qPCR was performed exerting TaqManUniversal PCR Master Mix (Thermo Fisher Scientific) in the ABI 7500HT real-time PCR system (Applied Biosystems). Calculation of relative expression was via the standard 2^-∆∆ct^ method. Adoption of glyceraldehyde-3-phosphate dehydrogenase (GAPDH) or U6 small nuclear RNA (U6 snRNA) was as loading controls for mRNA and miRNA, respectively. Primer sequences are presented in Table 1.

### 2.7. Western Blot

Extraction of total protein was with Radioimmunoprecipitation assay lysis buffer (Beyotime, China) in the light of manufacturer's instructions. Examination of protein concentrations was via the bicinchoninic acid protein assay kit (Thermo Fisher Scientific, Waltham, MA, USA). Separation of samples covering the identical amount of protein extraction was on 10% sodium dodecyl sulfate-polyacrylamide gel electrophoresis, and electroblot was done onto the polyvinylidene fluoride membrane (Millipore, USA). Block of the membrane was with 5% skim milk, and then addition was with primary antibodies CTSB (ab58802, 1 : 1000, Abcam), p-pi3k (4228, 1 : 1000, Cell Signaling Technology), p-AKT (4060,1 : 1000, Cell Signaling Technology), and GAPDH (AB8245, 1 : 1000, Abcam) for incubation. After a rinse in Tris buffered saline twine, incubation of the membrane was with horseradish peroxidase-conjugated secondary antibodies (1 : 1000, Abcam). Blots were developed adopting electrogenerated chemiluminescence substrates (Thermo Fisher Scientific), and analysis was performed adopting Image *J* software.

### 2.8. Luciferase Activity Assay

To verify the targeting of miR-183-5p with CTSB, a CTSB 3′' untranslated region fragment with wild-type (WT) or mutant-type (MUT) miR-183-5p putative binding site was cloned via PCR. Insertion of the PCR products was into the pMir-Glo vector (synthesized via Shanghai GenePharma Co., Ltd.). Seeding of HEK293 cells was into 96-well plates at a density of 1 × 10^5^ cells/well. Then, cotransfection of miR-183-5p mimic, mimic NC, and luciferase reporter vector was into HEK293 cells, respectively, adopting Lipofectamine 2000. After transfection of 24 h, successive measurement of the luciferase activity of the firefly and the kidney was performed adopting the Dual Glo luciferase detection system (Promega).

### 2.9. RNA Immunoprecipitation (RIP)

After collecting cells, lysis was with lysis buffer. Incubation of the supernatant from cell lysates was with human *anti*-Ago2 antibodies (SCBT, Santa Cruz, CA, USA) or NC antibodies (mouse immunoglobulin *G*, SCBT, Santa Cruz, CA, USA). Detachment of proteins was with proteinase K buffer, and detection of coprecipitated RNA was performed adopting the quantitative real-time PCR. Total RNAs were considered as input control.

### 2.10. Statistical Analysis

Processing of all data was performed adopting SPSS 21.0 statistical software (SPSS, Inc, Chicago, IL, USA). Manifestation of measurement data was in the form of mean ± standard deviation (SD). The two-group comparison was implemented adopting the independent sample *t*-test. Comparisons among multiple groups should be performed exerting one-way analysis of variance (ANOVA) and Tukey's post hoc test. Comparison of data among groups at different time points was implemented adopting repeated measures of ANOVA and the Bonferroni post hoc test. *P* < 0.05 was accepted as indicative of significant differences.

## 3. Results

### 3.1. Cur Constrains Inflammatory Response of Sepsis Mice and Strengthens Its Immune Function

To explore the action of Cur on LPS-stimulated sepsis mice, mice were given 20 mg/kg Cur in gavage for 3 d, and then intraperitoneal injection of LPS (10 mg/kg) was to stimulate the model of sepsis mice. In this study, functional changes in critical organs were observed. AST, ALT, BUN, and creatinine were considered as critical functional markers of the liver and kidney, separately. AST, ALT, BUN, and creatinine in the serum was detected, clarifying that AST, ALT, BUN, and creatinine were elevated in the LPS, while they were declined in the Cur (Figure 1(a)). The contents of TNF-*α*, IL-1*β*, and IL-6 in serum of the LPS were augmented, while the content of inflammatory factors was declined in the Cur (Figure 1(b)). Determination of the percentage of CD39^+^ Tregs in the tail venous blood was performed. The percentage of CD39^+^ Tregs in the LPS was observed to be distinctly elevated; nevertheless, it was declined with Cur treatment (Figure 1(c)). Histological evaluation was performed after gaining tissue. Adoption of liver and kidney tissue sections (*n* = 6) was for histological assessment (200 ×). Glomerular injury, dilatation of renal tubules, inflammatory cell infiltration, and vascular congestion in mice in the LPS were presented, which testified distinct injury of the renal tubule and liver. Cur treatment ameliorated these injuries (Figure 1(d)). The apoptosis index of liver and kidney tissues of mice in the LPS was elevated, and Cur treatment declined the apoptosis index (Figure 1(e)). These results illuminated that Cur was provided with the protection on the liver and kidney of sepsis mice. Above all, to explore whether miR-183-5p was boosted via Cur in the model of LPS-stimulated sepsis mice, measurement of miR-183-5p was performed. miR-183-5p was discovered to be silenced in sepsis mice. Nevertheless, Cur was still available to turn around this situation (Figure 1(f)). Consequently, the results elaborated the Cur restrained inflammatory response and strengthened the immune function in sepsis mice, and this process was nearly linked with the augment of miR-183-5p.

### 3.2. Elevated miR-183-5p Is Available to Further Accelerate the Protection of Cur

To further figure out the role of miR-183-5p in sepsis mice, sepsis mice were given 20 mg/kg Cur in gavage for 3 d before modeling, and injection of agomir NC or miR-183-5p agomir (10 nM per 20 g weight) was into the tail vein. The successful injection was verified (Figure 2(a)). The determination of serum biochemical indexes manifested AST, ALT, BUN, and creatinine in the serum were declined after elevating miR-183-5p (Figure 2(b)), and the contents of inflammatory factors (TNF-*α*, IL-1*β*, IL-6) were reduced (Figure 2(c)). Augmented miR-183-5p was available to decline the percentage of CD39^+^ Tregs (Figure 2(d)). Elevated miR-183-5p was available to ameliorate tissue damage and reduce apoptosis index (Figure 2(e) and 2(f)). To sum up, elevated miR-183-5p was available to further boost the protection of Cur.

### 3.3. MiR-183-5p Negatively Targets CTSB

To further explore the latent downstream mechanism of Cur of exerting the role via augmenting miR-183-5p, Starbase database predicted miR-183-5p was provided with the binding site with CTSB (Figure 3(a)). Subsequently, detection of CTSB in sepsis mice was implemented, illuminating that CTSB was augmented in sepsis mice, while Cur treatment was available to constrain CTSB (Figure 3(b)). Additionally, CTSB was distinctly declined after elevating miR-183-5p (Figure 3(c)). To further verify their targeting, the luciferase activity assay was carried out. The results illuminated cotransfection with CTSB-WT and miR-183-5p mimic was available to distinctively reduce the luciferase activity of cells (Figure 3(d)). The experiment clarified miR-183-5p and CTSB were crucially abundant in Ago2 immunoprecipitation (Figure 3(e)). All in all, miR-183-5p negatively targeted CTSB.

### 3.4. Silenced CTSB Is Available to Further Boost the Protection of Cur

To further explore the action of CTSB in sepsis mice, sepsis mice were given 20 mg/kg Cur in gavage for 3 d before modeling, and injection of si-NC or si-CTSB (10 nM per 20 g weight) was into the tail vein. The successful injection was verified (Figure 4(a)). The results of serum biochemical indexes clarified after silencing CTSB, AST, ALT, BUN and creatinine were declined (Figure 4(b)), and the contents of inflammatory factors (TNF-*α*, IL-1*β*, IL-6) were reduced (Figure 4(c)). Silence of CTSB was available to lessen the percentage of CD39^+^ Tregs (Figure 4(d)). Additionally, declined CTSB was available to ameliorate tissue damage and reduce apoptosis index (Figures 4(e) and 4(f)). In general, silence of CTSB was available to further boost the protection of Cur.

### 3.5. Cur Mediates the PI3K/AKT Pathway via miR-183-5p/CTSB Axis

The PI3K/AKT pathway exerts a crucial action in various functions of modulating cells (metabolism, growth, proliferation, survival, transcription, and protein synthesis). Studies have manifested helix B-surface peptide alleviated LPS-stimulated AKI and ameliorated renal function in sepsis rats via activating the PI3K/AKT pathway [19].

Detection of PI3K/AKT pathway was performed, clarifying that p-PI3K and p-AKT were distinctly declined in the LPS. The p-PI3K and p-AKT were crucially elevated after Cur treatment. After elevating miR-183-5p or silencing CTSB, p-PI3K and p-AKT were critically augmented (Figure 5). In brief, Cur mediated the PI3K/AKT pathway via the miR-183-5p/CTSB axis.

The western blot test of p-PI3K and p-AKT. The data in the figure are all measurement data, and each value represents the mean ± SD of six individuals.  ^*∗*^vs. the Sham, *P* < 0.05; ^#^vs. the LPS, *P* < 0.05; vs. the agomir NC, *P* < 0.05; $ vs. the si-NC, *P* < 0.05.

## 4. Discussion

As reported, Treg exerts a critical role in sustaining immune homeostasis, and CD39, an exonucleotide enzyme of hydrolytic proinflammatory ATP, is considered as a functional cell marker of Treg [20]. Antecedent studies have illuminated Tregs implicates in the pathogenesis of sepsis via stimulating immunosuppression [21]. Presently, numerous evidences elaborated that Cur is available to strengthen the suppression function of Treg in sepsis and sepsis-triggered acute organ dysfunction [22]. Nevertheless, the precise mechanism is unknown. Hence, this study was performed. It was founded that Cur treatment crucially declined AST, ALT, BUN, and creatinine in the serum of sepsis mice, reduced the content of inflammatory factors, and declined the percentage of CD39^+^ Tregs. Additionally, kidney and liver injury of mice were ameliorated as well, and the apoptosis index of the liver and kidney tissue was declined. These results elaborated that Cur was provided with the protection on sepsis mice.

Multiple researches have illuminated that LPS is the extremely mighty proinflammatory factors, being available to stimulate inflammatory responses after inhalation or systemic administration, and being appropriate for constructing the model of sepsis mice [23]. Consequently, in this study, Cur was administered initially, and then intraperitoneal injection of LPS was to stimulate the model of sepsis mice. Foregoing studies that have illuminated sepsis not only causes systemic and uncontrolled immune activation but also results in multiple organ failures, among which the liver and kidney are the extremely susceptible organs [24]. AST, ALT, BUN, and creatinine were the critical functional markers of the liver and kidney, separately. Consequently, in this research, detection of these indexes in sepsis mice with different treatments was to analyze the function of Cur in sepsis mice. It was discovered that AST, ALT, BUN, and creatinine in serum of mice, inflammatory factors like TNF-*α*, IL-1*β*, and IL-6, and the percentage of CD39^+^ Tregs were elevated after treatment with Cur [25]. Additionally, LPS treatment stimulated glomerular injury, dilatation of renal tubules, inflammatory cell infiltration, and vascular congestion in mice, and it also elevated the apoptosis index of liver and kidney tissues. These data testified the successful establishment of LPS-induced sepsis mice model. While Cur treatment critically turned around the action of LPS. Interestingly, it was discovered that Cur therapy critically elevated miR-183-5p. After further experiments, it was testified that Cur exerted an *anti*-inflammatory role in sepsis mice via augmenting miR-183-5p [26].

In this study, it was initially discovered that miR-183-5p was silenced in LPS-stimulated sepsis mice, while augmented miR-183-5p reduced AST, ALT, BUN, and creatinine in serum of sepsis mice, the content of inflammatory factors, and the percentage of CD39^+^ Tregs, and tissue damage was ameliorated and the apoptosis index declined. These data clarified that miR-183-5p was available to be adopted as a novel molecular diagnostic marker for sepsis, and augmented miR-183-5p was provided with a latent therapeutic value for sepsis mice [27]. Additionally, it was verified that the downstream target of miR-183-5p was CTSB.

CTSB, a lysosomal cysteine protease located in the extracellular space between keratinocytes, is available to modulate multiple physiological processes [28]. Though the role of CTSB in solid tumors has been completely certified, its up-regulation is nearly associated with tumor's progression [29]. Nevertheless, little is known about its action in other illnesses, especially sepsis. In this research, it was discovered that CTSB was elevated in sepsis mice, and silence of CTSB further boosted the protection of Cur. A foregoing study has illuminated that CTSB is linked with the PI3K/AKT pathway [30]. As reported, that PI3K/AKT signal transduction is a critical pathway for cell survival and proliferation, exerting a critical action in modulating the immune response and the release of inflammatory factor *in vivo* and *in vitro* via mediating the activation of downstream signaling molecules and participating in the occurrence and development of sepsis [31]. Consequently, the impact of sepsis on PI3K/AKT pathway was further explored. The results manifested that LPS critically declined p-PI3K and p-AKT, while p-PI3K and p-AKT were distinctively augmented after Cur treatment. Additionally, elevation of miR-183-5p or silence of CTSB distinctively augmented p-PI3K and p-AKT. These results illuminated that Cur mediated the PI3K/AKT pathway via the miR-183-5p/CTSB axis in sepsis mice [29, 30, 31].

## 5. Conclusions

1. The histological evaluation of liver and kidney sections (*n* = 6) of experimental mice (200 ×). LPS can cause glomerular injury, renal tubular dilatation, inflammatory cell infiltration, and vascular congestion in mice, indicating that LPS has obvious damage to the kidney and liver of mice, and the apoptotic index of liver and kidney tissue in LPS mice is increased; Cur treatment improved these injuries and reduced the apoptosis index.
2. Cur treatment increased mir-183-5p *in vivo*. Experiments showed that Cur played an *anti*-inflammatory role in sepsis mice by enhancing mir-183-5p.
3. The experiments uncover a brand-new latent mechanism of Cur in sepsis, that is, Cur elevated miR-183-5p via CTSB-mediated PI3K/AKT pathway to strengthen the LPS-stimulated immune function of sepsis mice. The study offers a theoretical foundation for Curcumin as a novel treatment for sepsis.

## Figures and Tables

**Figure 1:** Cur constrains the inflammatory response of sepsis mice and strengthens its immune function. (a) AST, ALT, BUN, and creatinine in the serum; (b) contents of inflammatory factors (TNF-*α*, IL-1*β*, IL-6); (c) flow cytometry detection of percentage of CD39^+^ Tregs; (d) HE staining test of glomerular injury, dilatation of renal tubules, inflammatory cell infiltration, and vascular congestion in mice; (e) TUNEL staining detection of the apoptosis index of the liver and kidney tissue in mice; (f) RT-qPCR examination of miR-183-5p. The data in the figure are all measurement data, and each value represents the mean ± SD of 6 mice.  ^*∗*^vs. the Sham, (P) < 0.05; ^#^vs. the LPS, (P) < 0.05.

**Figure 2:** Elevated miR-183-5p is available to further boost the protection of Cur. (a) RT-qPCR test of miR-183-5p; (b) AST, ALT, BUN, and creatinine in the serum; (c) contents of inflammatory factors (TNF-*α*, IL-1*β*, IL-6); (d) flow cytometry test of percentage of CD39^+^ Tregs; (e) HE staining examination of tissue injury; (f) TUNEL staining test of apoptosis index. The data in the figure are all measurement data, and each value represents the mean ± SD of six individuals.  ^*∗*^vs. the agomir NC, (P) < 0.05.

**Figure 3:** MiR-183-5p negatively modulates CTSB. (a) Starbase database prediction of the binding site of miR-183-5p with CTSB; (b-c) RT-qPCR and western blot detection of CTSB; (d) the luciferase activity assay verification of the targeting of miR-183-5p with CTSB; (e) RIP experiment validation of the targeting of miR-183-5p with CTSB. The data in the figure are all measurement data, and each value represents the mean ± SD of 6 individuals.  ^*∗*^Vs. the Sham, (P) < 0.05; ^#^vs. the LPS, (P) < 0.05; vs. the agomir NC, (P) < 0.05.

**Figure 4:** Silence of CTSB is available to further boost the protection of Cur. (a) RT-qPCR and western blot detection of CTSB; (b) AST, ALT, BUN, and creatinine in the serum; (c) contents of inflammatory factors (TNF-*α*, IL-1*β*, IL-6); (d) flow cytometry test of percentage of CD39 + Tregs; (e) HE staining examination of tissue injury; (f) TUNEL staining detection of apoptosis indexes. The data in the figure are all measurement data, and each value represents the mean ± SD of 6 individuals.  ^*∗*^vs. the si-NC, (P) < 0.05.

**Figure 5:** Cur mediates the PI3K/AKT pathway via the miR-183-5p/CTSB axis.

**Table 1:** RT-qPCR primers.

Genes	Primer sequences (5′'– 3′')
MiR-183-5p	F : CGCGGTATGGCACTGGTAGA
	R : AGTGCAGGGTCCGAGGTATTC

CTSB	F : CACTGACTGGGGTGACAATG
	R : CACTGACTGGGGTGACAATG

U6	F : CTCGCTTCGGCAGCACA
	R : AACGCTTCACGAATTTGCGT

GAPDH	F : CGGAGTCAACGGATTTGGTCGTAT
	R : AGCCTTCTCCATGGTGGTGAAGAC

## Data Availability

The figures and tables used to support the findings of this study are included in the article.
